The article "Concepts and Application of DNA Origami and DNA Self-Assembly: A Systematic Review" was published in 2021. Journal: Appl Bionics Biomech.

# Concepts and Application of DNA Origami and DNA Self-Assembly: A Systematic Review

**DOI:** 10.1155/2021/9112407

**Published:** 2021-11-16

**Authors:** Wei Liu, Huaichuan Duan, Derong Zhang, Xun Zhang, Qing Luo, Tao Xie, Hailian Yan, Lianxin Peng, Yichen Hu, Li Liang, Gang Zhao, Zhenjian Xie, Jianping Hu

**Affiliations:** ^1^Key Laboratory of Coarse Cereal Processing, Ministry of Agriculture and Rural Affairs, School of Pharmacy, Sichuan Industrial Institute of Antibiotics, Chengdu University, Chengdu 610106, China; ^2^School of Marxism, Chengdu Vocational & Technical College of Industry, Chengdu 610081, China

## Abstract

With the arrival of the post-Moore Era, the development of traditional silicon-based computers has reached the limit, and it is urgent to develop new computing technology to meet the needs of science and life. DNA computing has become an essential branch and research hotspot of new computer technology because of its powerful parallel computing capability and excellent data storage capability. Due to good biocompatibility and programmability properties, DNA molecules have been widely used to construct novel self-assembled structures. In this review, DNA origami is briefly introduced firstly. Then, the applications of DNA self-assembly in material physics, biogenetics, medicine, and other fields are described in detail, which will aid the development of DNA computational model in the future.

## 1. Introduction

As the most core issue in the field of science and technology, the computational problem has become an important indicator to evaluate the advanced degree of science, engineering, equipment, and technology [1]. At present, high-performance computing has been widely used in aerospace, meteorology, biological information processing, and other fields [2, 3], playing an increasingly important role in the national economy and social life. Computer is one of the three major scientific revolutions in the 20th century, which has made great contributions to the development of computing theories such as graph theory and operations research [4]. In the past decade, nontraditional computing, including artificial neural network computers, quantum computers, optical computers, nanometer computers, and molecular biological computers [5–7], has developed rapidly and been adopted by more and more scholars. Given the advantages of ultra-large-scale parallelism and huge data storage capacity, natural computing based on DNA pairing has become one of the main development directions of nontraditional high-performance computing [8, 9].

In 1994, Professor Adleman [7] proposed DNA computing and successfully solved the Hamilton path problem. Different from electronic computer based on the principle of Turing machine, DNA computing is a new information processing model based on biochemical reaction mechanism. The basic idea of DNA computing is to encode information using the unique double helix structure of DNA molecules and the Watson-Crick [10] principle of base complementarities, so as to obtain all possible solutions to mathematical problems. Specifically, the information from the original question is mapped into DNA double strands according to specific rules, in other words, and different DNA sequences are used to encode information under the effect of related biological enzymes and finally generate various data pools. The mapped molecular chains are then developed into new DNA strands through controlled biochemical operations, providing all possible solutions to the original problem. Finally, molecular biological detection technology is used to extract the required new molecular chains to solve the practical problems [11].  Figure 1 shows how to obtain the shortest route from city A through 6 cities and back to city A using traditional genetic algorithm and DNA calculation. As shown in Figure 1, DNA computing not only solved the problems of actual biochemical reactions efficiently but also greatly reduced calculation time by avoiding the recursion and iteration process in genetic algorithm calculation. The specific combination of bases makes DNA computing predictable, and the diverse structure of DNA nanomolecules can be easily characterized. DNA molecule has become a kind of biological self-assembled material, which is characterized by its stability, easy to be synthesized, easy to be modified, and good biocompatibility [12].

In the 1980s, Seeman [13] proposed that the regular periodic structure formed by DNA base complementation could be used to establish the framework structure of proteins or other molecular crystals, thus providing an ideal research tool for crystallography. In recent years, DNA self-assembly technology has developed rapidly. According to the strict complementary base pairing principle, it takes DNA molecule as the basic material and spontaneously forms a highly organized, highly ordered, structured, functional, information-based, life-related complex [14]. Notably, the novel DNA self-assembly strategy-DNA origami combines a long single strand of DNA with a series of designed short DNA fragments by complementary base pairs to create highly complex nanostructures in a controlled way. It has already played an important role in the fields of biophysics, materials science, biology, bionics, gene analysis, molecular recognition, cellular medicine, and biological imaging [15]. This review first provides the definition and research background of DNA module, then describes the theory and application of DNA origami, and finally introduces the wide application of DNA self-assembly in life science in detail (Figure 2).

## 2. Background of DNA Self-Assembly Modules

As a carrier of genetic information, DNA is responsible for the synthesis of RNA and proteins in organisms, which are both material basis for growth, replication, response to the environment, and life basis needed for eukaryotic cells to develop from fertilized eggs into mature organisms [16, 17]. It was first discovered in cell nucleus in 1869 and was identified as genetic material by the pneumococcal transformation experiment in 1944 [18, 19]. By the mid-1940s, it became clear that DNA was composed of three parts: phosphoric acid and deoxyribose and nitrogen-containing bases, the latter of which contains adenine (A), guanine (G), cytosine (C), and thymine (T) bases [20]. In 1953, Watson and Crick discovered that DNA is a double helix structure formed by alternating deoxyribose and phosphoric acid connected by ester bonds [10]. X-ray diffraction shows that the paired bases always appear in fixed combinations (i.e., A and T, G, and C) [21].

Based on the principle of base complementary pairing, single strands of DNA can not only hybridize with each other but also recognize other DNA strands in parallel. Two patterns of DNA recognition can be present in the same solution simultaneously, thus providing a natural parallel computing tool. Besides, the sequence of DNA bases provides a good means of storing and encoding large amounts of information. Previous studies have found that the data storage capacity per gram of DNA reaches 215 PB, equivalent to that of 220,000 1 TB hard drives [22]. Furthermore, DNA has two advantages as a storage medium: (1) it can be made into any desired shape; (2) it has a storage half-life of thousands of years [23, 24].

Given the uniqueness and applicability of DNA, how to detect and read its stored information are also a hot research issue. From the 1960s to 1970s, agar gel electrophoresis was used as a primary tool for nucleic acid analysis, which can observe and determine the size of DNA molecules [25]. In the mid-1970s, Sanger sequencing [26], a more accurate method of determining nucleotide sequence, laid a foundation for further molecular biology studies to obtain the target DNA fragment. In the 1980s, gene chips [27] based on the principle of hybridization sequence were used to detect DNA fragments containing specific sequences. Similarly, the electrochemical chip method based on this principle also detects biomarkers through electrical signals, focuses on the difference between single-stranded with double-stranded DNA, and achieves accurate and rapid sequencing. During the 1990s, Binning [28] introduced a more powerful tool—atomic force microscope (AFM)—for understanding the microscopic world, which has become an important tool for studying the structure and function of DNA. Based on AFM, the structure of three-dimensional cyclic DNA molecules can be observed in various environments by providing local charge density and physical properties of biomolecules; the interaction forces between biomacromolecule receptors and ligands can be measured; receptor or ligand molecules can be personalized stretched.

With the development of DNA research, its uniqueness, nomenclature, and complementary base pairing have attracted extensive attention in various scientific fields. In 1994, computer scientist Aldeman [29] introduced the idea of using bioindustrial technology to solve complex mathematical problems and opened up a new research field (i.e., DNA computing) based on the parallelism of base complementary pairing [30]. In general, DNA computing can be divided into intramolecular, intermolecular, and supramolecular categories in essence [31]: intramolecular computation mainly relies on morphology transformation and the construction of programmable state machine based on a single DNA molecule; intermolecular computing focuses on hybridization between different DNA molecules; supramolecular computing involves the self-assembly process of original DNA molecules with different sequences [29, 32]. There are three stages in DNA computing: (1) the test tube stage: verifying the feasibility of the DNA calculation principle based on a solution reaction; (2) the surface stage: as a transition stage, DNA molecules are fixed to a solid surface, overcoming operational difficulties and preventing them from being lost in the test tube; (3) the stage of DNA chip towards maturity and application: a large amount of genetic information can be rapidly monitored and efficiently analyzed using hybridization sequence [33, 34].

As an emerging field, DNA computing plays a vital role in data encryption, intelligent control, biological chemistry, combinatorial chemistry, medicine, data flow logic operations, Boolean circuit simulation, and so on [35, 36]. In 1995, Winfree et al. proposed the DNA self-assembly technology by combining DNA calculation with Tile theory and developed the software capable of simulating self-assembly behavior in 1998 [30, 37]. In fact, the emergence of DNA self-assembly has led the development direction of DNA computing. Self-assembly is a common process, which is defined as an orderly structure formed spontaneously by basic units under certain conditions. The biomacromolecular self-assembly is mainly driven by noncovalent bond forces including Coulomb force, van der Waals force, hydrophobic force, stacking force, hydrogen bond, and base stacking. DNA self-assembly technology is a procedure of continuous self-correction and self-improvement from simple to complex, from disorder to order, and from multicomponent convergence to a single component [38, 39]. Besides, base complementary pairing is the basic principle of DNA self-assembly, ensuring a high degree of selectivity, constant specificity of intermolecular interactions, and predictability of product structure.

In 1964, Holliday proposed the Holliday models [40] to explain homologous recombination, which significantly stimulated research inspiration of DNA self-assembly technology. In 1983, Seeman's group [13] summarized the stable structure of Holliday junctions through experiments and verified the branched DNA structure formed by electrophoresis and UV detection, laying the structural foundation for the assembly of more complex DNA structures. On the basis of Holliday model, Winfree et al. [30] wound different DNA strands into two rows to construct two DX modules (i.e., DAE and DAO), which could form a large area of two-dimensional DNA structure (see Figure 3). The DAE module has two different kinds of sticky ends, through which DNA can be extended horizontally and vertically to obtain more complex basic modules (1) and (2), then forming a larger two-dimensional DNA structure through noncovalently bonds [41, 42]. In 2000, La Bean [43] reported another new DNA self-assembly module—the TX module—in which the DNA strands were wound into three rows. Compared with DX, the TX module increases structural gap and provides more space to accommodate other molecules, facilitating the assembly of more complex molecules. It is worth mentioning that in 2003, Yan [44] extended a new crossmodule on the basis of the TX module, which further expanded the space for embedding molecules.

With the further research on these DNA self-assembly modular structures, a variety of simple graphic structures (such as two-dimensional array, square grid, and polyhedron) can be obtained through combination and assembly [45]. Due to the limitation that size and shape are difficult to precisely control, extremely complex polymer structures cannot be obtained only through the most basic modular assembly of DNA. In 2006, a new DNA self-assembly method, DNA origami, was proposed by Rothemund [46]. According to the concept of DNA origami, a series of symmetrical DNA patterns such as squares and stars can be constructed by repeatedly folding the long strand of natural DNA single strand and fixing it with the short strand (also known as staple chain) [44]. Compared with the traditional bottom-up assembly method, DNA origami has a series of obvious advantages: accurate assembly and arrangement on the nanometer scale, the availability of more complex and fine structure, ordinary experimental conditions, simple operation techniques, high assembly efficiency and strong fault tolerance, etc. In 2010, Wang et al. [47] found that in addition to hydrogen bond between complementary bases, the base stacking force can also be used to assemble DNA structures. By adjusting base stacking force, Rothemund et al. successfully gained a large-sized two-dimensional DNA nanostructure [48].

In addition to DNA origami, dynamic DNA self-assembly is also a commonly mentioned and adopted strategy for the construction nanostructure models. It can achieve the artificial control on different nanoscale structures and conformation conversion by designing DNA sequences or changing the environment. According to the transformation mechanism, dynamic DNA self-assembly can be divided into two categories: environment change-driven and strand substitution change-driven [49–51].

## 3. Theoretical Extension of DNA Origami

With the development of society and the continuous progress of science and technology, the bottom-up DNA self-assembly method rather than the top-down micromachines can meet the increasing needs of computational model complexity [12, 52]. As an outstanding DNA self-assembly module, DNA origami has a broad application prospect. Specifically, DNA origami can be used to construct the most complex and refined two-dimensional DNA nanostructures, which subsequently serve as a template to assemble functional nanomaterials or molecules. The implementation of DNA origami consists of the following four steps: (1) DNA double helix skeleton chains are arranged in parallel, and the overall outline is similar to origami structure; (2) designing the crossover structure; (3) adding a large number of “staple” chains; and (4) the self-assembly of the skeleton chains and the staple chains is completed under annealing treatment in a specific salt (Figure 4(a)) [15, 53]. Based on DNA origami, many ingenious two-dimensional plane origami structure, including rectangle, square, five-pointed star, smiling face, map of China, and dolphin, have been constructed [46, 54, 55]. Moreover, DNA origami is also widely used in biomedicine, structural materials, molecular machines, biological computing, etc. [56–59]. Especially in the current era when DNA nanotechnology is combined with emerging artificial neural networks, artificial intelligence, big data storage, and large-scale parallel technology [60–62], DNA computing shows more unique advantages compared with traditional computing methods.

### 3.1. DNA Origami and Super Origami

In contrast to the strict modular assembly, DNA origami has no special requirements for the stoichiometric ratio between long strands and complementary staple strands. In fact, excessive staple chains can reduce the probability of mismatch, improve the efficiency of self-assembly, and finally enable the synthesis of high-quality DNA self-assembly structures. In other words, sufficient staple chains can provide many templates and carriers for the continuous and efficient reassembly of other functional nanoparticles after a series of reactions. Objectively, DNA origami also has some disadvantages. Due to the limitation of the length of the long DNA strand, the size of the two-dimensional nanostructure assembled by DNA origami is only about 100 nm, making it impossible to assemble a larger structure [58, 63, 64]; DNA origami structure is potentially unstable due to the influence of environmental conditions, such as pH values, chemical properties, and temperature [65, 66]. Later, by combining DNA origami with traditional self-assembly methods, scientists used origami structure as the basic self-assembled structural unit to gain a larger hierarchical structure. In 2010, Liu et al. [67] acquired a vertically intersecting structure with DNA origami, which then grew to a large two-dimensional structure in both directions through the hierarchical assembly.

In 2011, Zhao et al. [59] proposed a new assembly method-super origami (i.e., Origami of Origami). They first synthesized two-dimensional origami structural units with the basic DNA origami module, then reassembled nanostructure units through bridge strand, and finally obtained larger DNA origami structures. Subsequently, Yang et al. [68] adopted a more extensive double-stranded DNA as an origami template and constructed a larger DNA nanostructure by adjusting the assembly conditions. The successful assembly of larger-sized DNA origami structures has a significant impact on the field of DNA self-assembly and nanodevice research.

### 3.2. A Carrier for Nanoparticle Assembly

DNA origami structure can be used as a carrier to accurately arrange nanoparticles [69, 70]. By adjusting the coupling effect of nanoparticles, DNA origami structure serves as a substrate to construct semiconductor nanocrystals with special optical and electronic properties [71–73]. In general, the local field effect is significantly enhanced when the spacing of gold nanoparticles is less than 10 nm [74]. According to the spatial positioning of DNA origami, Ding et al. accurately assembled gold nanoparticles with different sizes onto the surface of origami structure and precisely controlled the spacing within 10 nm [75]. According to Shen's work, the DNA nanotube carrier was gradually combined with the gold nanoparticles embedded in DNA sequence to obtain the optically active DNA tubular structure [76, 77]. It is worth mentioning that this tubular structure has an obvious circular dichroic signal at the plasmon resonance wavelength of nanogold, which has been successfully adopted by optical waveguides, detectors, etc.

Apart from gold nanospheres, one-dimensional nanomaterials have tremendous applications in many various fields due to their more substantial Raman enhancement effect and plasmon resonance effect [78, 79]. Nevertheless, the one-dimensional structure of gold nanorods has a high degree of freedom, which increases the complexity of the assembly process. Moreover, due to the randomness and uncontrollability of the arrangement and assembly of such structures, it will be difficult to accurately control the accumulation of gold nanorods, which greatly impedes the further application of gold nanorods [80]. In 2011, Pal [81] designed and synthesized triangular DNA origami structures with specific capture strands, which was precisely recognized by the gold nanorods modified with sulfhydryl single-stranded DNA through complementary base pairing. In the resulting gold nanorods, parameters such as order, distance, and angle can be precisely manipulated. In the subsequent synthesis of plasma nanomaterials, by adjusting the coupling degree of plasma field, changing the resonance effect of plasma particles, improving the local field strength, and so on, the unique optical and electromagnetic properties were obtained.

### 3.3. Nanoscale DNA Chips

With the development of microelectronics technology, computer chips with higher and higher integration have more and more demanding requirements on the size of components. However, the working principle and process technology of the devices are not conductive to the manufacture of microchips. At present, the biggest difficulties in microchip manufacturing are as follows: (1) with the increase of the number of stacked layers, the probability of circuit mismatch in the process will be higher; (2) as the device size decreases, some of its electrical properties decline, which requires a new device design. As a new nanoself-assembly method, DNA origami has the unique advantages of large storage capacity, low energy consumption, and high parallelism, which has great potential application value in the preparation of nanodevices.

In 2009, IBM and Rothemund [82] etched the binding sites of origami structures on inorganic materials' substrates (such as silica and diamond) by electron beam etching and dry oxidation etching. Then, using DNA molecules as the architectural frame, they designed a precise arrangement pattern through deposition and self-assembly, resulting in a controllable and ordered origami structure on the surface of the inorganic semiconductor material. The strategy that combines DNA origami with nanolithography has made it possible to make tiny nanoscale computer chips. Similarly, Hung et al. assembled gold nanoparticles with DNA origami structures in two steps: (1) etching origami structural adsorption sites on inorganic material substrates through electron beam etching [83]; (2) depositing an origami structure on the substrate and getting a large area of repeating unit structure. In general, the effective combination of “top-down” electron beam etching [84] and “bottom-up” DNA origami makes DNA origami nanostructures have great development potential and extensive application prospects in many nanometer fields such as nanometer devices and nanometer materials.

## 4. Application of DNA Self-Assemble

DNA folding and DNA assembly are closely related. DNA folding, as the premise of DNA assembly, lays a theoretical foundation for DNA assembly, while DNA assembly, as a result of DNA folding, plays an important role in various fields. With the continuous development of DNA module and origami technology, DNA self-assembly has shown an immeasurable application prospect in the fields of biophysics, bionics, biological imaging, genetic analysis, and drug delivery. Specifically, in material physics, DNA nanostructure serves as a physical carrier to composite various materials to form nanoclusters. In the field of biogenetics, DNA nanostructure is widely used in bionics, nucleic acid analysis, gene analysis, and other scientific researches. While in the medical field, DNA nanomachines are mainly involved in the following aspects: as a drug carrier to achieve the specific delivery of drugs within the cell and solving the problem of accurate microscopic imaging in vivo by specific recognition with fluorescent labeled DNA.

### 4.1. As a Biophysical Tool

Due to the structural design ability and dynamic controllability of DNA self-assembly technology, DNA nanotechnology has been widely used in biophysics, especially in the study of single-molecule systems. In 2008, Rinker first used DNA nanostructures as scaffolds to control the interactions of multicomponent biomolecules and studied the distance effect of aptamer binding to bivalent proteins at the single-molecule level [85]. Inside the cell or on a protein surface, DNA self-assembly technology was also used to explain the conformational change of molecular motors caused by the energy conversion from hydrolysis of adenosine triphosphate into mechanical energy [86–88]. In eukaryotic cells, cytoplasmic dynein and kinesin-1 both are molecular motors that can move freely in microtubules and transport some endogenous substrates; the polarities of dynein and kinesin are opposites, moving towards the positive and negative poles of microtubules, respectively; substrate transportation requires the simultaneous action of the two molecular motors. The Reck-Peterson group first constructed immobilized substrates using 12 double helix structures [89, 90]. By studying molecular motor complexes with different polarities, they found that the main factor determining the direction of substrate transportation was the ratio of cytoplasmic dynein to kinesin 1 [91, 92].

The emergence of DNA origami mentioned above has solved the problem of accurately controlling the composite of nanomaterials at the nanoscale [93]. Through simple DNA double helix strands, metal nanoparticles can be organized and arranged, and more complex nanomaterials can be constructed by using addressable DNA origami structures [94–96]. Yan et al. accurately controlled the number and position of gold nanoparticles on the triangular origami by adjusting the size, distance, and angle of the particles in an orderly manner [75]. Acuna et al. studied the distance between a single fluorescent gene and a quenched gene using gold nanoparticles [97]. Taking advantage of the accuracy and specificity of DNA origami, Zhao and Shen also trapped nanoparticles of different sizes at specific locations [98, 99]. Gang constructed an octahedral DNA origami structure with gold nanoparticles attached to each vertex, and the origami-gold nanoparticle complex could then be assembled into a larger ordered crystal structure [100]. In addition to nanoparticles, single-layer carbon nanotube structures can also be precisely arranged. Maune et al. fixed carbon nanotubes onto the surface of DNA origami structure through a series of chain substitution reactions [101]. It was also replicated in the experiment of Zhao and Mangalum, demonstrating that carbon nanotubes can be arranged in a predesigned direction and position [102–104].

### 4.2. Applications in Bionics

Due to the complexity of biological systems, it is difficult to study many scientific problems and phenomena at the single-molecule level, including nucleic acid analysis, motile protein movement, mechanism of action of biological enzymes, and nanopore sensing [105]. With the programmability of DNA self-assembly technology, a biomimetic system and even a complete artificial cell can be constructed, possessing most of the function of normal cell. In biomembrane systems, the phospholipid bilayer is responsible for ion transport and biomolecular exchange, regulated by physical or chemical stimulation of nanopores. This process involves the production of energy and the synthesis of proteins, which are very important for sustaining life [106]. At present, solid nanopores [107] and composite DNA nanopore channels [108] both have been successfully constructed and used to explore their recognition patterns and transport mechanisms.

As an emerging nanopore structure, composite DNA nanopore channels have the advantages of better stability, reversibility, elastic properties, and more manageable adjusting pore size [109]. Different DNA origami cannot be distinguished at the same temperature, salt concentration, and pH value, but can be separated from solid nanopores under a specific voltage applied.

Combining two-dimensional DNA origami structure with nanoscale solid nanopore, the Keyser group obtained the first DNA origami-solid composite nanopore channel structure under the condition of ensuring small pore size and stable origami channel, which was applied in the detection of SSDNA, dsDNA, proteins, and other biological molecules [110]. Subsequently, a variety of composite DNA nanopore channels have been constructed. Simmel et al. used DNA nanostructures as components to construct transmembrane channels within the phospholipid bilayer, which can successfully distinguish the single DNA molecules with different properties through single-channel electrophysiological experiments. Similarly, based on the DNA tile structure, a channel that can carry cholesterol molecules through the lipid membrane was designed [111]. Krishnan et al. reported a group of DNA origami nanopore structures with stable electrical conductivity [112]. Farimani et al. synthesized a DNA origami-graphene hybrid nanopore structures that can distinguish four types of DNA bases [113].

### 4.3. Application in Biological Imaging

Biological imaging is an important research method to understand organism structure and to elucidate physiological functions, by obtaining microstructural images of biological cells and tissues directly through optical or electron microscopy [114–116]. With the development of the digital imaging technique and computer image analysis technology, as well as the emergence of new fluorescent probes, advanced lasers and highly sensitive photodetectors, three types of super-resolution microscopic imaging methods have been proposed. The first is a laser scanning imaging method based on point spread function (PSF). The representative technology is stimulated emission depletion of radiation (STED), which shows the advantages of better resolution and faster speed, as well as the disadvantage of greater light damage to the sample [117, 118]. The second is a wide field imaging method based on Laser & Photonics Reviews (LPR), and the representative technique is structure illumination microscopy (SIM) with fast imaging speed but low resolution [119]. The third is the most commonly used method, single-molecule localization (SML), and the representative techniques are photoactivation localization microscopy (PALM) [120] and stochastic optical reconstruction microscopy (STORM) with high imaging accuracy [121]. However, the use of this method requires the solution of the technical bottleneck in molecular fluorescence labeling, namely, how to program fluorescent molecular interactions to enhance the specificity of fluorescent molecules.

Based on the programmable and specificity of DNA hybridization, Professor Jungmann developed the DNA-PAINT technology, which is simpler and more straightforward than conventional DNA self-assembly operations [122]. In DNA-PAINT, the random fluorescent switch is dominated by a repetitive and transient binding-dissociation effect between the oligonucleotide chains labeled with a fluorescent molecule (imager chain) and the complementary docking chain on the DNA nanostructure. For the unbound state, only the partially quenched imager chains can produce a background fluorescence signal; when the imager chain and the docking chain are combined, the fluorescence emission signal can be detected by total internal reflection fluorescence microscopy (TIRF) or highly inclined and laminated optical sheet (HILO) [123]. At present, this technique has been adopted by multicolor super-resolution imaging (~25 nm) of DNA nanostructures [124]. In 2017, Jungmann et al. upgraded the DNA-PAINT technology to 2D/3D multicolor super-resolution imaging by combining the docking chain with antibodies [125]. Using the programmability of DNA molecules and Exchange-PAINT technology, they immobilized cellular protein components and achieved continuous multiple imaging with sub-10 lateral resolution in vitro. In addition, they obtained for the first time 10-color super-resolution results of DNA nanostructures in vitro, achieving the 4-color imaging and three-dimensional 3-color imaging of immobilized cellular protein targets.

There are two methods to construct imaging probes using DNA self-assembled structures to encode fluorescence molecules. The first method is to encode fluorescence molecules according to their intensity. Luo introduced the fluorescent molecules into the DNA dendritic structure (Figure 5(a)) and accurately controlled the number of different fluorescent molecules in the probe [126]. Two common fluorescent molecules were combined with a color probe with various fluorescent signals to achieve the simultaneous detection of multiple target DNA. The method is straightforward to encode and read signal, but has the disadvantage of fewer fluorescent probes encoded. By binding three fluorescent molecules to a DNA six-spiral tubes with length of 800 nm, Yin made 216 fluorescent probes (Figure 5(b)), which could be accurately distinguished under TIRF [124]. With the help of this probe, in situ imaging of Candida albicans surface antigens was achieved. Another way is to encode fluorescence molecules according to their position, including two subclasses of reaction specificity and location specificity. Hao et al. [127] first introduced three kinds of ligands that specifically respond to pH, Hg^2+^, and ATP into a DNA tetrahedron, then used the allosteric effect of DNA tetrahedron to observe the change of optical signals, and finally achieved the accurate imaging of these targets (Figure 5(c)). Given the characteristic that DNA origami would accumulate in the kidney after metabolism, the imaging therapy was successfully achieved on mice with acute kidney injury [29, 128] (Figure 5(d)).

### 4.4. Application in Genetic Analysis

As functional fragments of DNA molecules and genetic information material, genes play an irreplaceable role in predictive medicine, disease prevention, health management, personalized medical services, etc. [129–132]. Since 2008, DNA self-assembly technology has been widely applied to the detection of RNA molecules. Ke et al. [133] synthesized a specific sequence of nanoprobe and attached them onto DNA origami, forming rigid V-shaped structures with specific RNA molecules. With AFM imaging, the height of the V-shaped structure can be observed to determine whether the probe has bonded to the corresponding RNA molecule. Due to electrostatic repulsion and steric effect, the hybridization distribution between the probe chain and the origami was not uniform, and the hybridization efficiency of the probe near the edge was relatively highest. In order to enhance this phenomenon and reduce steric hindrance noiset, Fan et al. changed the original V-shaped probe into a simple linear probe [134].

This “sandwich” framework (i.e., origami-probe-RNA) can also be hybridized with longer target DNA, making it a potential universal platform for DNA detection. Based on this platform, single-base polymorphism (SNP) genotyping can be achieved through chain substitution reaction. Seeman et al. visualized a single SNP site and the SNP site of a diploid heterozygote. They also found that the entirely complementary target DNA strand could replace the extracted strand; if the DNA strands are not completely complementary, the signal molecules will be quenched [135]. On the basis of the original classical chain substitution reaction, Yin et al. used a new probe to study the single base differentiation under different experimental conditions based on toehold-mediated strand displacement reaction, which is very important for biomedical research and clinical applications [136]. Zhang et al. utilized a toehold-based strand displacement and introduced a fluorescent DNA probe to distinguish the polymorphism of a single base on a target DNA sequence [137]. Fluorescence quenching molecules and toehold chains both were modified by double-stranded fluorescent probe at both ends, and the complementary toehold region (where chain replacement reaction takes place) was connected to the target DNA sequence. It is worth noting that the probe will emit a fluorescent signal if the target DNA is completely complementary, and not vice versa. In addition, there are some limitations in the application of chain displacement reactions: the target DNA needs to be processed to ensure that it is utterly complementary to the extracted DNA strand; it is impossible to directly detect long fragment sequences.

### 4.5. Application in Cell Drug Delivery

As a new mode of biological drug delivery, cell drug delivery can effectively avoid the risks of adverse reactions, too large fluctuation of blood concentration, and rapid degradation of genetic drugs [138]. Due to molecular designability and membrane permeability, DNA self-assembled structures can be used as drug carriers. DNA nanostructures can interact with a variety of functional molecules through changes in shape and size, covalent bonding, nucleic acid base pairing, biotin-avidin reaction, intercalation, aptamer-ligand reaction, and DNA-protein reaction, all of which support their important role in cell drug delivery [139–141]. In addition, DNA nanostructures have the addressability and can precisely control the location of drug-delivery molecules, presenting advantages different from inorganic and organic nanomaterials [142].

In addition to biocompatibility, degradability, and specificity, DNA nanostructures are also characterized by low toxicity and high stability, which have been widely used in the targeted transport of anticancer drugs to suppress the expression of tumor cells [143–145]. Based on DNA origami, Douglas et al. constructed a hexagonal cross-section barrel structure that could carry gold nanoparticles or Fab fragments (Figure 6(a)) [146]. Fu et al. used Douglas's structure to load anticancer drugs and accurately transported them to the testing target, effectively inhibiting the growth of cancer cells (Figure 6(b)) [147]. Up to now, many potent anticarcinogenic drug molecules, including doxorubicin and CpG oligonucleotides, have been successfully loaded into DNA nanostructures with better clinical performance [143]. Li et al. constructed a DNA origami tetrahedral structure carrying CpG oligonucleotide drugs into macrophage RAW264.7, which was recognized by TLR9 to produce an apparent immune stimulus response [148]. With the help of the same tetrahedral structure, siRNA was delivered in vivo to inhibit the expression of tumor-related genes [149]. Similarly, Xia et al. constructed functional nanostructures by coupling doxorubicin and peptide, which effectively improved the drug uptake rate of malignant glioma cells U87MG [150].

It is important to note that manipulating DN nanomachines in living cells also presents several challenges: (1) the components of DNA nanomachines, including motion orbits, must be stably absorbed by cells without rejection; (2) DNA nanomachines need to be driven from the offstate to the onstate by specific active molecules; and (3) the autonomous movement of DNA nanomachines in living cells requires self-powered and monitored in real-time. Chris et al. constructed a novel DNA nanomachine that successfully overcame the above challenges and entered living cells through endocytosis [151]. Thus, it is increasingly possible for drug-loaded nanomachines to target and kill tumor cells without damaging healthy tissue. In 2016, Sylvain Martel et al. developed a nanorobot imitating magnetotactic/aerotactic bacteria, which was driven by bacteria flagella to complete drug transportation (Figure 6(c)) [152]. Recently, the Zhao group constructed a DNA rectangular origami in M13 phage and produced a tubular nanomachine by linking thrombin (Figure 6(d)) [153]. As the tube-shaped nanomachines bound to the nucleoli of tumor blood vessel cells, a special protein on the cell surface would activate the nanomachines to release antitumor drugs. Remarkably, this experiment not only presented promising results in vivo but also did not elicit any significant immune response.

## 5. Conclusion

This review first introduces the definition of DNA module, the theory, and development status of DNA origami, followed by a detailed description of the application of DNA self-assembly technology in various fields of natural science, especially in the field of biomedical. With the development of DNA computing, DNA self-assembly structures with different shapes and functions have been successfully constructed, but there are still six challenges in DNA self-assembly technology: (1) there is no unified DNA computer model to solve all kinds of problems; (2) encoding affects the quality of hybridization and ultimately determines the feasibility and speed of DNA computing; (3) detection of solutions is an important problem in DNA computing research, closely related to the calculation results; (4) DNA self-assembly technology has developed to the level of arbitrary complex three-dimensional shapes, while most of computational systems can only deal with two-dimensional DNA origami structure; (5) there are some errors in the existing DNA recombination technology, and the catalytic efficiency of enzymes cannot reach 100%, which will affect the efficiency and reliability of DNA calculation; and (6) although DNA computing has the unique advantage of simulating a wide range of physiological environments (i.e., different temperatures, enzymes, and pH values), the stability of the calculations remains a challenge.

In view of the limitations of DNA self-assembly mentioned above, it is necessary to focus on coding research, build a computing system with general functions, and effectively solve detection problems. In addition, constraints should be added to the coding design to reduce the range of error, and finally, a DNA self-assembly structure computing system with strong environmental adaptability is developed. It is believed that with the further development of DNA self-assembly technology, intelligent control at the atomic level will be achieved in the future, which will bring breakthroughs in the fields of material physics, biogenetics, and medicine. Simultaneously, some nontheoretical prospects should be concerned: we believe that DNA self-assembly in the future should be interwoven with some more disciplines and blossom in more fields. Besides DNA, can amino acids also be incorporated into the system? Can unique amino acid structures act as bridges between DNA links through various interactions?

## Figures and Tables

**Figure 1:** The shortest route from city A through B, C, D, E, F, G, and then back to city A is calculated by DNA algorithm and genetic algorithm.

**Figure 2:** The process and characteristics of applying DNA algorithm and genetic algorithm to nanomaterials, biomedical medicine, chip, artificial intelligence, and other applications.

**Figure 3:** The process of the two-dimension structures constructed by DAE and DAO modules.

**Figure 4:** Principles of DNA origami (a) and two-dimensional AFM imaging structures including Chinese map (b), pentacle, and smiley face (c) [46, 55].

**Figure 5:** The imaging probe was constructed according to the intensity (a, b) and position (c, d) of fluorescence molecules. [124, 126–128].

**Figure 6:** Applications of DNA nanostructures in cell drug delivery [146, 147, 152, 153].
